# Technical and Biological Complications of Screw-Retained (CAD/CAM) Monolithic and Partial Veneer Zirconia for Fixed Dental Prostheses on Posterior Implants Using a Digital Workflow: A 3-Year Cross-Sectional Retrospective Study

**DOI:** 10.1155/2021/5581435

**Published:** 2021-07-06

**Authors:** Paolo De Angelis, Giulio Gasparini, Francesca Camodeca, Silvio De Angelis, Margherita Giorgia Liguori, Edoardo Rella, Francesca Cannata, Antonio D'Addona, Paolo Francesco Manicone

**Affiliations:** ^1^Department of Head and Neck and Sensory Organs, Division of Oral Surgery and Implantology, Fondazione Policlinico Universitario A. Gemelli IRCCS—Università Cattolica del Sacro Cuore, Rome, Italy; ^2^Department of Head and Neck and Sensory Organs, Division of Oral and Maxillo-Facial Surgery, Fondazione Policlinico Universitario A. Gemelli IRCCS—Università Cattolica del Sacro Cuore, Rome, Italy; ^3^Private Practice, Ascoli Piceno, Italy

## Abstract

**Objective:**

The introduction of CAD/CAM and the development of zirconia-based restorations have allowed clinicians to use less expensive materials and faster manufacturing procedures. The purpose of the study was to analyze the differences, in terms of mechanical and biological complication, in multiunit zirconia fixed dental prosthesis (FPDs) on posterior implants produced using a digital workflow. *Method and Materials*. This study was a retrospective investigation, and patients treated with screw-retained monolithic or partial veneer FPDs on dental implants were selected. Periapical radiographs were taken at baseline and at the 3-year follow-up. Complications were recorded and classified as technical and biological ones.

**Results:**

The study population included 25 patients. The occlusal and interproximal corrections were not clinically significant. In the study sample, the survival rate and success rate of the FPDs after 3 years were 100% and 96%, respectively. One implant failed immediately after placement.

**Conclusion:**

Monolithic zirconia FPDs and partial veneer FPDs showed a 100% survival rate, presenting an interesting alternative to metal ceramic restorations. The partial veneer FPDs had a higher technical complication rate than the monolithic FPDs; however, no statistically significant difference was found.

## 1. Introduction

Over the years, a variety of new digital technologies and restorative materials for implant-supported prostheses have been developed [1]. Metal–ceramic restorations, which can be produced using several alloys, made using a traditional approach based on conventional impressions, stone casts, and the lost-wax technique, have long-term data and are considered the gold standard in fixed prosthodontics [2–5]. However, this approach has some disadvantages, such as its high cost, the time-consuming nature of the procedure due to the analogic method of fabrication, interoperator variability, and finally, limited esthetics [6].

The introduction of computer-aided design/manufacturing (CAD/CAM) allowed clinicians to use cheaper materials and faster manufacturing procedures, increasing the efficiency of the prosthetic treatments [3]. The development of this technology led to precisely designed virtual prosthetic devices that can be predictably fabricated in a highly automated manner, standardizing the quality of the products [7–9]. Furthermore, patients' esthetic expectations and preference for ceramic restorations have led to the progressive replacement of metal–ceramic restorations [10]. Beyond esthetics, the other advantages of implant-supported ceramic restorations include a reduction in bacterial and plaque adhesion [11], better marginal integration between crowns and abutments, prevention of soft tissue inflammation [12–16], and uniform thickness of the cementation space [17–19].

Accordingly, zirconia-based restorations have become a popular choice in implant dentistry thanks to its mechanical properties such as high flexural strength and the unique crack-inhibitory material properties of yttria-stabilized tetragonal zirconium dioxide polycrystals (3Y-TZP) [20, 21], as well as its natural inclusion in a digital workflow [5].

However, conventional 3Y-TZP zirconia is too opaque for monolithic restorations because of its high internal light scattering [22, 23]. Therefore, to overcome this esthetic limit, zirconia-based restorations are veneered with ceramic, but this has been associated with complications such as porcelain chipping [5].

Recently, changes in composition, structure, and production methods have led to the development of more translucent types of monolithic zirconia, reducing the need for veneering and ensuring higher biocompatibility, higher esthetics, and better biomechanical properties than traditional materials [24]. Thus, it is possible to increase the optical properties of zirconia, making them similar to that of other ceramics, while minimizing the possibilities of fracture or chipping thanks to the monolithic nature of the prostheses [25].

Therefore, the purpose of this retrospective clinical study was to analyze the clinical outcomes of multiunit zirconia FPDs on posterior implants produced using a digital workflow.

## 2. Materials and Methods

A total of 25 patients who received screw-retained monolithic or partial veneer FPDs on dental implants between January 1, 2016, and January 1, 2017, were selected for this cross-sectional study.

All procedures took place at a private dental practice in Ascoli Piceno, Italy. All procedures were performed according to the Declaration of Helsinki guidelines on experimentation involving human subjects. Each participant enrolled in the study received explanations on the study design and objectives and provided written informed consent.

Due to the retrospective nature of this study, it was granted an exemption in writing by the local ethics committee.

Patients satisfying the following inclusion criteria were selected for the study:

1. Patients treated with an implant-supported FPD to rehabilitate a Kennedy Class II
2. Age ≥ 18 years
3. Type 3 implant placement (from 3 to 4 months of healing after extraction)
4. Presence of antagonist's teeth (either natural or restored)
5. Sufficient mesiodistal and interocclusal space
6. At least 3 years of follow-up

The exclusion criteria were as follows:

1. Untreated periodontitis
2. No residual keratinized tissue at experimental area
3. Diagnosis of temporomandibular joint disorders assessed using the Diagnostic Criteria for Temporomandibular Disorders (DC/TMD) [26]
4. Systemic diseases that could hamper normal healing processes
5. Smoking
6. Excessive alcohol consumption
7. An American Society of Anesthesiologists physical status classification of ≥III

From an initial sample of 32 eligible patients, 7 patients did not complete the three-year follow-up; therefore, 25 patients constituted the study sample.

The decision as to which of the two protocols to perform was made after a discussion with the patient, explaining the advantages and disadvantages as well as the cost of each treatment.

Patients' charts were obtained, and data (such as age, sex, date of implant placement and prosthesis delivery, presence of bruxism, number and type of complications, and esthetic outcomes) were extracted.

Prosthesis delivery was considered as baseline. All rehabilitations were carried out by the same trained clinician and dental technician.

### 2.1. Treatment Protocol

A complete periodontal examination and a preoperative CBCT were performed to complete the surgical and prosthetic planning. The presence of bruxism was also assessed preoperatively following the bruxism's international consensus definition [27].

Implant fixtures (Straumann Dental Implant System, Straumann AG, Basel, Switzerland) were placed under local anesthesia, according to the manufacturer's guidelines. Preoperative prosthetic digital planning was performed for all cases, and when indicated, a guided surgery approach was used to facilitate the positioning of the access holes in the preferred areas (Figures 1–3). After 3 months, implant stability was clinically investigated by visual inspection and tactile sensation when removing the healing component before the digital impression was taken using an intraoral scanner and following the manufacturer recommendations (CEREC AC Omnicam, Sirona Dental Systems GmbH, Bensheim, Germany). Color assessment was done during the same appointment to provide the information required by the dental lab technician to fabricate the final restoration with a shade guide (Vitapan 3D-Master, Vita Zahnfabrik, Bad Sackingen, Germany), a shade light (Demetron Shade Light, Kerr Corporation, Orange, CA, USA) and digital photography.

The dental technician used a software program (Dental CAD, EGSolutions; Heraus Kulzer GmbH, Hanau, Germany) to design and fabricate each FPD. During the FPD design and the digital modelling, a minimum of 0.5 mm thickness for the monolithic zirconia was observed in all areas; also, the minimum connector dimension was set at 12 mm^2^, while interproximal and occlusal contact tightness at 0.10 mm.

Full-contoured prostheses were made of acrylic resin and tried in intraorally.

The adopted CAD/CAM monolithic zirconia (Biodynamic Multilayer 1200/600 Mpa Progressive, Biodynamic Dental, Correggio, Italy) is a material that presents higher flexural strength in the cervical region (1200 MPa), where more mechanical strength is needed, and lower flexural strength (600 MPa) in the incisal region, where more translucency is preferred. Zirconia was milled (CORiTEC 250i, imes-icore GmbH, Eiterfeld, Germany), and then, monolithic restorations were infiltrated with the brush infiltration technique (H2O Colors, Biodynamic Dental, Correggio, Italy). The infiltrated FPDs were dried thoroughly before sintering.

Partial veneer zirconia restorations were designed digitally with a cut-back procedure of 0.4 mm to provide adequate space for the veneering in the buccal surfaces of the zirconia frameworks. Anatomic reduction was performed only in the regions without occlusal contacts. The FPDs were manually veneered using ceramic veneer (Art Oral ZR, REOX, Mestre, Italy) and finally stained and glazed.

All FPDs were bonded to the metal substructures with an adhesive luting composite resin (Multilink Hybrid Abutment; Ivoclar Vivadent AG, Schaan, Liechtenstein) following the manufacturer's guidelines to obtain one-piece hybrid cement-screw-retained FPDs. The passive fit of the FPDs was checked intraorally using the Sheffield test. Interproximal contact tightness was evaluated intraorally by assessing the resistance to the passage of dental floss (0.05 mm width × 0.004 mm height; Oral-B). Occlusion was evaluated with shimstock foil.

When required, adjustments were performed using ceramic-specific diamond rotary instruments while being water-cooled and then polished (SHOFU polishing kit, Shofu Inc., Kyoto, Japan). All FPDs were inserted and screwed in with a manual torque control ratchet at 35 Ncm. The retorque application after 10 minutes was used to increase the screw loosening torque. The screw access holes were closed using polytetrafluoroethylene tape and composite resin (Figures 4 and 5).

The interproximal contact tightness was evaluated at delivery by assessing the resistance to the passage of dental floss (0.05 mm width × 0.004 mm height; Oral-B, Procter & Gamble, Cincinnati, Ohio), and the occlusion was assessed with shimstock foil. During prosthetic placement, any interproximal or occlusal surface adjustment was recorded with a score ranging from 1 to 3. The occlusal surface adjustment was based on the analysis of the area after the occlusal registration with a 40 *μ* articulating paper using a two-tone representation of static and dynamic occlusion (1 = no correction required; 2 = minimal correction required; 3 = significant correction required) [2]. After the appropriate correction, the restoration was properly polished to remove any monoclinic phase produced by the adjustments [28].

The interproximal contact adjustment was based on the resistance to the passage of dental floss (1 = mild resistance; 2 = moderate resistance; 3 = severe resistance).

The esthetic of the restoration was then analyzed with the white esthetic score (WES) [29].

The patients were visited as part of their standard follow-up after 1 week and every 6 months from the prosthesis delivery. At these appointments, if deemed necessary, an ultrasonic supragingival debridement procedure was undertaken.

During the 1-, 2-, and 3-year follow-ups, the following peri-implant parameters were measured with a UNC-15 periodontal probe:

- *Bleeding On Probing (BOP)*. At six sites (mesiobuccal, midbuccal, distobuccal, distolingual, midlingual, mesiolingual) of each implant
- *Probing Pocket Depths (PPD)*. At six sites (mesiobuccal, midbuccal, distobuccal, distolingual, midlingual, mesiolingual) of each implant

Peri-implant parameters were recorded by a single clinician (P.D.A.).

Periapical radiographs were taken with the long cone parallel technique at baseline (prosthesis delivery) and at the 3-year follow-up. A silicone bite was placed in the holding system, allowing precise repositioning during each follow-up visit. The magnification factor was measured on each radiograph by dividing the known diameter of the implant with the diameter measured on the radiograph. Linear measurements (mm) on the digital images were performed to record the distances of the most coronal points in the mesial and distal ridge aspects from the implant shoulder and were then adjusted by the magnification factor.

Also, at the 3-year follow-up, the full-mouth plaque score (FMPS) and the full-mouth bleeding score (FMBS) were measured.

The survival and success rates of the prosthesis were assessed; the survival indicated whether the FPDs were physically in the mouth, while the success was defined as the absence of any complications. Complications were classified as mechanical/technical and biological ones.

Mechanical complications included the following:

- Fracture of an occlusal screw
- Loosening of an occlusal screw
- Loosening of an abutment
- Fracture of an abutment
- Fracture of an implant

Technical complications included the following:

- Loss of retention
- Fracture and/or chipping of ceramic
- Fracture of the framework

The technical complications were also classified as major, medium, and minor complications, as proposed by Lang et al. [30]. The major complications involved cases requiring replacement of the restoration, while abutment fracture, veneer, or framework fractures were considered medium complications; minor complications were those to be corrected with small efforts, such a small chipping. We also examined the opposing teeth and/or restorations to record complications that might be associated with the FPDs. The presence or absence of wear was also clinically evaluated using a 5× medical loupes. Patients were enrolled in a maintenance program which consisted in a clinical assessment of hygiene and occlusion performed yearly.

### 2.2. Statistical Analysis

The descriptive statistics used for the continuous factors included the mean, standard deviation (SD), and median; for categorical factors, absolute and relative frequencies (%) were utilized. The technical complication rate according to the presence of bruxism, type of opposing dentition, and the number of implants was analyzed with Fisher's exact test. The WES between monolithic and veneered restoration was compared with the Mann–Whitney *U* Test. All analyses were conducted using Stata (version 14.2, StataCorp, College Station, TX). Two-tailed probabilities are reported, and nominal statistical significance was defined using an observed significance level of 0.05.

## 3. Results

The study sample consisted of 25 patients (14 women and 11 men; mean age: 56.9 years, SD: 11 years). All participants received implant-supported FPD restoration; 14 FPDs were located in the upper jaw while 11 in the lower jaw. Eleven FPDs were porcelain-veneered (44%) while 14 FPDs were monolithic (56%). Eighteen FPDs were supported by two implants (72%) while seven FPDs were supported by three implants (28%). Thirteen FPDs (52%) had opposing natural dentitions while 12 (48%) had tooth- or implant-supported fixed prostheses. Two patients treated with veneered FPDs (18%) and four patients treated with monolithic restorations (29%) were affected by bruxism.  Table 1 summarizes the demographic data.

### 3.1. Technical Assessment

The occlusal and interproximal corrections at prosthesis delivery were not clinically significant, with a mean of 1.2 ± 0.5 for occlusal adjustments and a mean of 1.1 ± 0.3 for interproximal adjustments. Only two FPDs required mild interproximal corrections (8%), while three FPDs (12%) required occlusal corrections (two cases of mild corrections and one case of significant correction). At the end of the follow-up period, all FPDs were in use, and none had a major technical complication causing restoration failure. After 3 years of clinical service, the survival rate of the FPDs in the study sample was 100%. The only technical recorded for the FPDs was a case of ceramic chipping on the buccal cusp of the inferior first premolar (4%), in a patient affected by bruxism which occurred 31 months after prosthesis delivery in a partially veneered restoration, with natural dentition as the antagonist (Table 2). This was a repairable complication, and the FPD did not require replacing or any additional expense. The success rate of the FPDs was 96%.

Bruxism (*p* = 0.240), the presence of a partial veneer (*p* = 0.440), the type of opposing dentition (natural or restored) (*p* = 1), and the number of implants (2 or 3) (*p* = 0.280) had no statistically significant effect on the technical complication rate of the FPDs.

A case of opposing tooth fracture was recorded in a maxillary second premolar after 13 months, which was restored with root canal treatment and a single crown. At the 3-year follow-up, no wear of the restorations was observed using medical loupes and 5x magnification.

### 3.2. Biological Assessment

A total of 57 dental implants were evaluated, and only one implant failed, immediately after placement, resulting in a 3-year implant survival rate of 98%. After the follow-up period, 92% of the patients were free of any type of complications. At the 3-year follow-up, two patients had marginal bone loss of >1.5 mm, while the mean FMBS and FMPS were 22% and 17%, respectively.

### 3.3. Esthetic Assessment

A mean overall white esthetic score of 8.4 ± 0.9 was recorded, 8.8 ± 0.7 for the partial veneer FPDs, and 8.1 ± 0.9 for the monolithic FPDs. A higher mean esthetic score was recorded in the partial veneer FPDs, and there was a statistically significant difference (*p* = 0.039); however, the patients treated using monolithic zirconia had a clinically successful value in all cases treated.

## 4. Discussion

The purpose of the present investigation was to examine the clinical outcomes of monolithic or partial veneer zirconia for implant supported FPDs produced using a digital workflow.

The decision to use this restorative material was motivated by the growing demand for greater esthetics and lower costs and shorter production time while retaining high product quality and attempting to digitalize and standardize the procedure.

In a systematic review, Sailer et al. observed a 5-year survival rate of 98.7% for metal–ceramic FPDs supported by implants. However, the 5-year success rate was 84.9% [24]. The 5-year survival rate of zirconia FPDs (93.0%) was significantly lower than that of metal–ceramic FPDs. For both types of restorations, the predominant technical complication was chipping and/or fracture of the veneering ceramic [24, 25, 29–31].

According to Pjetursson et al., all-ceramic FPDs had a lower survival rate than metal–ceramic FPDs; however, no statistically significant differences were observed except for the glass-infiltrated alumina FPDs [32].

Furthermore, the meta-analysis of Lemos et al. recorded no statistically significant differences comparing different materials in terms of prosthesis survival rate as well as technical and biological complications [6]. However, the study mentioned that the short-term follow-up of the selected studies was a limitation [6]. In the present study, the survival and success rates were 100% and 96%, respectively, and there were no major technical complications necessitating replacement of the prosthesis.

Despite metal–ceramic restorations being considered the gold standard for many years [6], the choice of zirconia cores with or without veneering is becoming one of the most popular for restoring implant-supported prostheses today [22, 33].

In the present study, no catastrophic framework fractures occurred, which is in agreement with the results of Cheng et al., who demonstrated that the fracture strength of zirconia used for single crowns was sufficiently high for sustaining normal occlusal loading even if parafunctional patients were included in the study [34]. However, in another study, Cheng et al. noted that one FPD in a patient affected by bruxism fractured at the connector, outlining that FPDs, had higher complication rates than single crowns, although there was no statistically significant difference [35]. From a biomechanical point of view, zirconia frameworks have demonstrated favorable outcomes for implant-supported restorations, but it should be also noted that, to reduce the risk of framework fractures, there should be appropriate thickness with the necessary load-bearing capacity [36, 37]. In another study, Ozer et al. reported that monolithic zirconia with a thickness of 1.3 mm showed higher flexural strength than monolithic zirconia with a thickness 0.8 mm, and the difference was statistically significantly [37].

The most frequently reported technical/mechanical complication of veneered zirconia prostheses is minor chipping of the veneering porcelain [38–42]. Yet, chipping fracture may not be considered a real failure because it does not affect function and also may not compromise esthetics and often requires only finishing and polishing of the prosthesis without replacement [43]. In fact, Larsson et al. found that many patients were unaffected or unaware of it [20]. Here, the only minor complication we encountered was a case of minor chipping in a veneered zirconia FPD (4%). This complication occurred in a patient with bruxism, indicating that bruxism may represent a risk factor for chipping, as reported by Kolgeci et al. [10]. For this reason, in patients considered at risk, the use of zirconia in monolithic restoration could avoid the unwanted complication of chipping [23]. The use of monolithic restorations may also be indicated in patients with an unfavorable occlusion, affected by parafunctions or with a fracture history, as well as in those cases where there is a limited space for restorative materials [23].

In the present study, there were no cases of fractures in the monolithic zirconia FPDs, in line with other studies [44, 45].

According to our results, monolithic FPDs showed a lower rate of technical complications and had only a slight inferior esthetic result; we therefore advise for clinicians to limit veneered restorations to clinical cases where given the characteristics of adjacent teeth, or the patient's request, it is paramount to obtain a restoration with the highest esthetic capabilities, despite a lower mechanical resistance. In all other cases, a monolithic restoration can and will provide adequate esthetic results for a rehabilitation of a Kennedy Class 2, while at the same time reducing the risk of complications.

Another frequently reported minor complication for screw-retained FPDs is screw loosening, which did not occur in any of the patients in the present study. According to Kolgeci et al., screw loosening was a rare and clinically not significant event occurring only in the early phase of their follow-up [10]. However, this technical complication is considered frequent, as reported by Kreissl et al. [46] in whose study it had a cumulative incidence of 6.7% within 5 years, in agreement with the outcomes of Pjetursson et al., who reported in their meta-analysis a cumulative incidence of 5.8% after 5 years [47]. These results are higher than that of the present study, probably due to the longer follow-up (5 years).

With regard to biological complications, only one implant failed immediately after positioning, before being prosthetically loaded.

Therefore, after 3 years of follow-up, 92% of patients were free from any kind of complications.

Furthermore, monolithic and veneered zirconia not only present high mechanical performance but also remarkable esthetic capabilities [48]. A statistically significant difference was recorded for esthetics, with a greater mean esthetic score recorded in the patients treated with partial veneer zirconia, even if in all cases successful integration of the restoration was achieved and confirmed at the 3-year follow-up. As Schmitter also showed, esthetics is a fundamental aspect for evaluating the clinical performance for this type of prosthesis, and the present study recorded a very promising esthetic score for both monolithic and veneered restorations [49].

In addition, analysis of the results allowed us to determine that using CAD/CAM technology allowed precise design of prosthetic devices; in fact, no restoration required significant correction during the prosthesis delivery. Only two FPDs required mild interproximal corrections (8%), while three FPDs (12%) required occlusal corrections (two cases of mild corrections and one case of moderate correction).

Despite the promising results of implant-supported zirconia prostheses, the sample size of the present study is small; there was no control group, and follow-up was short-term. Therefore, long-term prospective clinical investigations with a larger population are still necessary for determining the clinical reliability and viability of CAD/CAM technology.

## 5. Conclusions

Within the limitations of the present study, monolithic zirconia FPDs and partial veneer FPDs showed a 100% survival rate after 3 years of follow-up, indicating that they are a promising alternative to metal–ceramic restorations. The partial veneer FPDs had a higher technical complication rate than monolithic FPDs; however, there was no statistically significant difference. Monolithic restorations, given their esthetic capabilities and lower rate of complication, are the most appropriate choice for a posterior restoration. Further clinical medium- and long-term outcomes are required to validate this choice of treatment.

## Figures and Tables

**Figure 1:** Preoperative digital planning.

**Figure 2:** Initial situation before the implant placement.

**Figure 3:** Implant placement.

**Figure 4:** Occlusal view of the restoration after the placement.

**Figure 5:** Extraoral view at the 3-year follow-up.

**Table 1:** Sociodemographic and baseline characteristics.

*N* of patients	25
Gender	
Male	11
Female	14
Age (years)	56.9 ± 11
Type of prosthesis	
Partially veneered	11 (44%)
Monolithic	14 (56%)
Number of implants	
2	18 (72%)
3	7 (28%)
Bruxism	
Yes	6 (24%)
No	19 (76%)
Opposing dentition	
Natural	13 (52%)
Restored	12 (48%)

**Table 2:** The relative frequencies of complications and the results of the esthetic evaluation conducted with the white esthetic score.

	Technical complications (%)	Mechanical complications (%)	Biological complication (%)	WES (mean ± SD)
Monolithic restorations	0%	0%	7%	8.1 ± 0.7
Partially veneered restorations	9%	0%	0%	8.8 ± 0.9^∗^

^∗^ *p* < 0.05 for the interclass comparison.

## Data Availability

The data of the manuscript are available from the authors on request. Dr. Paolo De Angelis should be contacted to receive them.
